The article "Baculovirus Vector-Mediated Transfer of Sodium Iodide Symporter and Plasminogen Kringle 5 Genes for Tumor Radioiodide Therapy" was published in 2014. Journal: PLoS One.

# Baculovirus Vector-Mediated Transfer of Sodium Iodide Symporter and Plasminogen Kringle 5 Genes for Tumor Radioiodide Therapy

**DOI:** 10.1371/journal.pone.0092326

**Published:** 2014-03-19

**Authors:** Min Zhang, Rui Guo, Shuo Shi, Yin Miao, Yifan Zhang, Biao Li

**Affiliations:** Department of Nuclear Medicine, Rui Jin Hospital, Shanghai Jiao Tong University School of Medicine, Shanghai, China; Wuhan Bioengineering Institute, China

## Abstract

**Background:**

Both tumor cells and their supporting endothelial cells should be considered for targeted cell killing when designing cancer treatments. Here we investigated the feasibility of combining radioiodide and antiangiogenic therapies after baculovirus-mediated transfer of genes encoding the sodium iodide symporter (NIS) and plasminogen kringle 5 (K5).

**Methods:**

A recombinant baculovirus containing the NIS gene under control of the human telomerase reverse transcriptase (hTERT) promoter and the K5 gene driven by the early growth response 1 (Egr1) promoter was developed. Dual-luciferase reporter assay was performed to confirm the activation of hTERT transcription. NIS and K5 gene expression were identified by Western blot and Real-Time PCR. Functional NIS activity in baculovirus-infected Hela cells was confirmed by the uptake of ^125^I and cytotoxicity of ^131^I. The apoptotic effect of ^131^I-induced K5 on baculovirus-infected human umbilical vein endothelial cells (HUVECs) was analyzed by a flow cytometry-based assay. In vivo, NIS reporter gene imaging and therapeutic experiments with ^131^I were performed. Finally, the microvessel density (MVD) in tumors after treatment was determined by CD31 immunostaining.

**Results:**

The activation of hTERT transcription was specifically up-regulated in tumor cells. NIS gene expression markedly increased in baculovirus-infected HeLa cells, but not in MRC5 cells. The Hela cells showed a significant increase of ^125^I uptake, which was inhibited by NaClO_4_, and a notably decreased cell survival rate by ^131^I treatment. Expression of the K5 gene induced by ^131^I was elevated in a dose- and time-dependent manner and resulted in the apoptosis of HUVECs. Furthermore, ^131^I SPECT imaging clearly showed cervical tumor xenografts infected with recombinant baculovirus. Following therapy, tumor growth was significantly retarded. CD31 immunostaining confirmed a significant decrease of MVD.

**Conclusion:**

The recombinant baculovirus supports a promising strategy of NIS-based raidoiodide therapy combined with K5-based antiangiogenic therapy by targeting both the tumor and its supporting vessels.

## Introduction

The cloning of the sodium iodide symporter (NIS) gene and subsequent studies of its properties have led to a new approach of targeted radioiodide therapy for malignant cancers. NIS is a membrane glycoprotein that mediates the active uptake of one iodide ion along with two sodium ions across the basolateral membrane of thyroid follicular cells [1]. The uptake of radioiodide can be achieved by expressing the NIS protein in tumor cells via vector-mediated gene transfer to destroy the tumor by emission of β rays from ^131^I [2]. Moreover, the NIS gene can be used as a reporter for noninvasive monitoring of the expression or therapeutic effect of a transgene by single photon emission computed tomography (SPECT) or positron emission tomography (PET) [3].

The article "Baculovirus Vector-Mediated Transfer of Sodium Iodide Symporter and Plasminogen Kringle 5 Genes for Tumor Radioiodide Therapy" was published in 2014. Journal: PLoS One.

Tumor-specific promoters are well-documented to be suitable for vector-induced gene therapy for cancers. Human telomerase reverse transcriptase (hTERT) is an important component of the telomerase which is highly active in the vast majority of malignant tumors but is inactive in most normal cells [4]. The transcriptional activity of the hTERT gene promoter also has been observed exclusively in telomerase-positive cells [5]. These observations have highlighted the potential of targeted transfer of genes for expression under the hTERT promoter [6].

Formation of new blood vessels in response to hypoxia is a fundamental event in the process of tumor growth and metastatic dissemination. Some studies have suggested that antiangiogenesis drugs can enhance the tumor response to radiotherapy [7] or radionuclide therapy [8]. Plasminogen, which contains five kringle domains, is the precursor protein of a group of angiogenic inhibitors (angiostatin consists of kringle domains 1–4). Kringle 5 (K5), with a low molecular weight of 14 kDa and low immunogenicity, exhibits the most potent antiangiogenic effect compared to other kringle domain fragments [9]. Recombinant human K5 has been shown to induce apoptosis in proliferating endothelial cells [10] and enhance the antitumor effect when combined with ionizing radiation [11].

Cells respond to ionizing radiation with the activation of certain immediate-early genes, including members of the jun/fos and early growth response gene families [12]. The Egr1 gene belongs to the family of Egr genes encoding immediate-early transcription factors. Transcriptional activation of the Egr1 gene can be regulated by ionizing radiation through the radiosensitive CArG [CC(A+T-rich)6GG] elements in the promoter region [13]. Previous studies have shown that the Egr1 promoter could be activated not only by external radiation [14] but also by internal radiation from radioisotopes such as ^67^Ga and ^131^I [15], [16]. These findings led us to explore the use of the Egr1 promoter to drive expression of therapeutic transgenes introduced into irradiated cells.

The article "Baculovirus Vector-Mediated Transfer of Sodium Iodide Symporter and Plasminogen Kringle 5 Genes for Tumor Radioiodide Therapy" was published in 2014. Journal: PLoS One.

The success of gene therapy will depend on gene transfer vectors that facilitate the expression of a therapeutic gene. Viral vectors are efficient tools for genetic modification of the majority of somatic cells in vitro and in vivo. The baculovirus vector system, derived from insect viruses, is known to possess several advantages compared with other viral vectors, including a large packaging capacity, wide host range and safety in mammalian cells. Thus it has been utilized as a new generation gene therapy vehicle [17].

In the present study, we constructed a recombinant baculovirus dual expression vector in which the NIS and K5 genes are driven by the hTERT and Egr1 promoters, respectively (Bac-hTERT-NIS-Egr1-K5). This recombinant baculovirus was used to infect both tumor cells and tumor endothelial cells and investigate the feasibility of a strategy combining NIS-based β radiation therapy and K5-based antiangiogenic therapy simultaneously induced by radioiodine.

## Materials and Methods

### Ethics statements

The study was approved by the institutional review board and the experimental animals centre of Rui Jin Hospital affiliated to Shanghai Jiao Tong University School of Medicine.

### Cell lines and cell cultures

Human cervical cancer cells (Hela), human lung adenocarcinoma cells (A549), human glioma cells (U87), human fetal lung fibroblast cells (MRC5) and human umbilical veins endothelial cells (HUVECs) obtained from the Chinese Academy of Sciences were maintained in Dulbecco's Modified Eagle's Medium (DMEM) supplemented with 10% fetal bovine serum (FBS), 100 U/mL penicillin and 100 μg/mL streptomycin and incubated with 5% CO_2_ atmosphere at 37°C.

### Transient transfection and reporter assay procedure

Cultured cells (Hela, A549, U87 and MRC5) were plated in 24-well cell culture plates at densities of 5×10^4^ cells/well 24 h before transfection. The experimental reporter plasmid expressing firefly luciferase, pGL3-hTERT-Luc (1 μg/well), was transfected using Lipofectamine 2000 (Invitrogen) in accordance with the manufacturer's instructions. The same amounts of pGL3-Basic or pGL3-Control plasmids (Promega) were also transfected as negative and positive controls, respectively. A plasmid expressing renilla luciferase (pRL-SV40) (Promega) (20 ng/well) was cotransfected for evaluating transfection efficiency.

Cells were incubated with 0.5 ml medium containing transfection mixture for 6 h, and medium was changed. Incubation was continued for an additional 18 h. Then, medium was discarded and cells were washed twice with PBS. Cells in each well were harvested for firefly luciferase and renilla luciferase assay. Two luciferase activities were sequentially determined by dual-luciferase reporter assay system (Promega). All data of firefly luciferase activity were corrected for renilla luciferase activity to account for variation in transfection efficiency and expressed as a percentage of results using the positive control. Each transfection was conducted in triplicate, and data represent the mean±sd.

The article "Baculovirus Vector-Mediated Transfer of Sodium Iodide Symporter and Plasminogen Kringle 5 Genes for Tumor Radioiodide Therapy" was published in 2014. Journal: PLoS One.

### Plasmid construction and generation of recombinant baculovirus

The pGL3-hTERT-Luc plasmid, carrying the luciferase gene driven by the hTERT promoter, was kindly provided by Nicol Keith (Glasgow University, Glasgow, UK). The pGL3-Egr1-Luc plasmid, containing the luciferase gene under the control of the Egr1 promoter, was a kind gift from Gerald Thiel (University of Saarland, Medical Center, Homburg, Germany). The pET22b-K5 plasmid (His-tagged) was constructed previously in our laboratory. The baculovirus-based pFastBac Dual expression vector was purchased from Invitrogen.

To generate the plasmid carrying the NIS gene driven by the hTERT promoter, the NIS gene and luciferase gene were excised from the pfastbac-CMV-NIS [18] and pGL3-hTERT-Luc plasmids, respectively, with restriction endonucleases Hind III and Xba I. The NIS gene fragment was ligated to the pGL3-hTERT vector using T4 DNA ligase, generating the pGL3-hTERT-NIS plasmid. Similarly, the K5 fragment gene was obtained by double restriction digestion of the pET22b-K5 plasmid with Bgl II and Hind III and cloned downstream of the Egr1 promoter in the pGL3 vector, resulting in the pGL3-Egr1-K5 plasmid.

To construct the baculovirus dual expression vector, Sal I and Hind III enzyme sites were introduced by PCR flanking the hTERT-NIS fragment in the pGL3 vector, and then the fragment was subcloned into the pFastBac Dual vector with the same restriction enzymes. Similarly, EcoR I and Kpn I restriction sites were introduced in order to subclone the Egr1-K5 fragment into the pFastBac Dual vector containing the hTERT-NIS fragment. The resulting plasmid construct, containing the NIS sequence and K5 respectively coupled to the hTERT and Egr1 promoters, was designated as pFastBac-hTERT-NIS-Egr1-K5 and confirmed by DNA sequencing. The recombinant baculovirus Bac-hTERT-NIS-Egr1-K5 was generated using the Bac-to-Bac system (Invitrogen) according to the manufacturer's instructions. A recombinant baculovirus expressing the NIS gene driven by the CMV promoter (Bac-CMV-NIS-Egr1-K5) was constructed as a positive control, while recombinant baculoviruses expressing only the NIS gene or K5 gene (Bac-hTERT-0-Egr1-K5 and Bac-hTERT-NIS-Egr1-0) were constructed as negative controls in this study.

The article "Baculovirus Vector-Mediated Transfer of Sodium Iodide Symporter and Plasminogen Kringle 5 Genes for Tumor Radioiodide Therapy" was published in 2014. Journal: PLoS One.

### Baculovirus infection and cell irradiation

Cultured cells (Hela, MRC5 or HUVEC) were seeded in 6-well plates with DMEM (10% FBS) at least 24 h before infection. After infection with the recombinant baculovirus at the multiplicity of infection (MOI) of 2, the cells were incubated for 6 h with PBS, which was then exchanged with DMEM (10% FBS) for an additional 18 h of incubation.

In addition, to determine the optimal conditions for expression of radio-inducible K5, Hela cells were further irradiated with Na^131^I (Shanghai Xinke) at varying doses (0, 0.5, 1, 5, 10 and 20 MBq/mL) for different times (0, 6, 12, 18, 24 and 30 h) beginning 24 h after incubation with the recombinant baculovirus. Finally, the optimal expression condition was applied to HUVECs.

### RNA extraction and quantitative real-time polymerase chain reaction (qRT-PCR)

Total RNA samples from Hela and MRC5 cells were extracted with the RNeasy Mini Kit (Qiagen) and reverse-transcribed into cDNA using the Superscript RT kit (Invitrogen). qRT-PCR was performed with the SYBR Premix Ex Taq kit (TaKaRa). The sequences of primers for NIS and glyceraldehyde-3-phosphate dehydrogenase (GAPDH) were as follows: NIS: 5′-GTACATTGTAGCCACGATGCTGTA-3′ (sense), 5′-CCGTGTAGAAGGTGCAGATAATTC-3′ (antisense); K5: 5′-GAAGAAGACTGTATGTTTGGGAATGG-3′ (sense), 5′-GTGGTGG TGGTGGTGGTGGGCCGCACACT-3′ (antisense); GAPDH: 5′-GTCAAGCTCATTTCCTGGTATGAC-3′ (sense), 5′-CTCTCTCTTCCTCTTGTGCTCTTG-3′ (antisense). The cycling conditions were 95°C for 10 s, 40 cycles at 95°C for 5 s, 60°C for 31 s, and one cycle of 95°C for 15 s, 60°C for 1 min, 95°C for 15 s. According to the manufacturer's protocol, NIS and K5 expression levels were normalized to that of the GAPDH endogenous reference as given by: F value  = 2^−ΔΔCt^ [19]. The qRT-PCR analysis was repeated three times to obtain the mean values for each specimen.

### Western blot analysis

Lysates of baculovirus-infected cells were prepared by standard methods. Western blot analysis was then performed by incubating the filter with mouse anti-NIS (1∶500; Millipore), anti-His-tag (1∶500; Abgent) or anti-GAPDH (1∶10000; Abgent) antibody in Tris-buffered saline Tween-20 overnight at 4°C, followed by incubation with peroxidase-conjugated goat anti-mouse immunoglobulin G (1∶2500; Santa Cruz Biotechnology) for 1 h at room temperature. Immunodetection was carried out using an ECL Western blot detection kit (Pierce).

### In vitro iodide uptake studies

Cells (5×10^4^) seeded in 24-well plates were infected with Bac-hTERT-NIS-Egr1-K5 (MOI of 2) for 24 h. After subsequent washing with buffered Hanks Balanced Salt Solution (bHBSS; supplemented with 10 μmol/l sodium iodide and buffered with HEPES, pH 7.3), the cells were incubated for 5∼120 min at 37°C with 0.5 mL of bHBSS containing 3.7 kBq Na^125^I (Shanghai Xinke) in the presence or absence of 30 μM NaClO_4_. At various time points, cells were washed twice with ice-cold bHBSS and lysed with 4 N NaOH. The radioactivity was measured using a γ-counter (Shanghai Rihuan). Bac-hTERT-0-Egr1-K5 was used as a negative control. All of the following experiments were performed in triplicate.

The article "Baculovirus Vector-Mediated Transfer of Sodium Iodide Symporter and Plasminogen Kringle 5 Genes for Tumor Radioiodide Therapy" was published in 2014. Journal: PLoS One.

### Cell proliferation assay

Cell proliferation was determined by using the cell counting kit-8 (CCK-8) with WST-8 dye (Beyotime Institute of Biotechnology) according to the manufacturer's instructions. Briefly, 5×10^3^ cells were seeded per well in a 96-well plate and divided into three groups (blank, Bac-hTERT-0-Egr1-K5 and Bac-hTERT-NIS-Egr1-K5), all of which were incubated for 18 h with Na^131^I at 5 MBq/mL. Subsequently, cells were washed with bHBSS and incubated in the presence of 10% FBS for 4 days. At the end of the incubation, 10 μL WST-8 dye was added to each well for incubation with the cells at 37°C for 1 h. Finally, the absorbance was determined at 450 nm using a microplate reader (Thermo). Cell survival was expressed as the percentage of absorbance to that of the blank group without ^131^I incubation. Data are represented as means ± standard deviation (SD).

### Apoptosis assay by flow cytometry

HUVECs were divided into three groups (blank, Bac-hTERT-NIS-Egr1-0 and Bac-hTERT-NIS-Egr1-K5), each incubated with 5 MBq/mL ^131^I for 18 h. Thereafter, the cells were trypsinized, centrifuged, aliquoted into tubes and labeled with Annexin V and propidum iodide (PI) using the FITC Annexin V Apoptosis Detection Kit (BD Pharmingen). Annexin V and PI stainings were performed following the manufacturer's recommendations. Flow cytometric analysis was performed using a Flow Cytometer (Becton Dickinson). Cells that stained FITC Annexin V positive and PI negative were considered to be in early apoptosis. The groups without incubation with ^131^I were used to define their basal levels of apoptosis. Percentages of early apoptotic cells in ^131^I-treated groups were then determined by subtracting the base apoptotic rate. All of the following experiments were performed in triplicate.

### In vivo tumor scintigraphic imaging and therapeutic experiments with ^131^I

Tumor xenograft models were generated by subcutaneous injection of viable Hela cells (5×10^6^ cells suspended in 150 μl PBS) into the right axilla of the mice. A 3-day pretreatment with Lugol's iodine solution (5 μl per mouse daily) by gavage was performed to reduce iodide uptake by the thyroid gland and maximize radioiodine uptake in the tumor.

The article "Baculovirus Vector-Mediated Transfer of Sodium Iodide Symporter and Plasminogen Kringle 5 Genes for Tumor Radioiodide Therapy" was published in 2014. Journal: PLoS One.

For imaging experiments, six mice were divided into two groups and injected intratumorally with 5×10^8^ plaque-forming units (pfu) of Bac-hTERT-NIS-Egr1-K5 and PBS, respectively. At 24 h after infection, mice were injected with 7.4 MBq of Na^131^I via the tail vein under isoflurane anesthesia. Tumor xenograft scingtigraphic imaging was performed using SPECT with a high-resolution pinhole collimator (GE Infinia) at 0.25, 0.5, 1, 2, 4 and 16 h post-injection. The total injected dose was also determined. After imaging, tumors were harvested and weighed. Regions of interest in the tumor were quantified and expressed as a fraction of the total amount of applied radioiodine per gram of tumor tissue (i.e., percentage injected dose per gram, %ID/g).

For ^131^I-mediated therapeutic experiments, mice were infected with 5×10^8^ pfu of Bac-hTERT-NIS-Egr1-K5, Bac-hTERT-0-Egr1-K5 or Bac-hTERT-NIS-Egr1-0. After 24 h, 37 MBq of Na^131^I was given to mice via the tail vein. PBS was also intratumorally injected in two control groups with or without ^131^I. Six mice were included in each group, and tumor volumes were followed for 15 days. At the end of the follow-up period, animals were anesthetized, and the tumors were removed and analyzed by immunohistology.

### Immunohistochemical staining of CD31 and determination of microvessel density (MVD)

Tumors were harvested in 4% paraformaldehyde for 24 h and embedded in paraffin. For immunostaining, 5-μm deparaffinized poly-L-lysine-coated sections were treated with 3% hydrogen peroxide for non-specific binding. A CD31 antibody (Santa Cruz Biotechnology) diluted at 1∶200 was used for immunohistochemical staining by the peroxidase-antiperoxidase technique. Brown staining indicated a positive result.

MVD was expressed as the number of microvessels per field. A single microvessel was defined as any CD31-immunostained endothelial cell that was separated from adjacent tumor cells and other connective tissue elements. Large vessels with thick muscular walls were not counted, and the presence of a lumen was not necessary for scoring as a microvessel. In each sample, the three most intense areas of neovascularization were identified and counted at low power (magnification, 100×). Average vessel counts of the three selected fields were recorded.

### Statistical analysis

Data were analyzed using the SPSS 13.0 software. Each experiment was carried out in triplicate, and results were calculated as means ± standard deviation (SD). Comparisons among experimental groups were performed using analysis of variance (ANOVA). P<0.05 was considered statistically significant.

## Results

### Transcriptional activity of hTERT promoter in tumor or normal cells

To confirm that the activation of hTERT transcription was up-regulated in telomerase-positive tumor cells but not in normal cells, a transient transfection of luciferase reporter plasmids was performed (Figure 1). The transcriptional activity of the positive control in each cell line was considered as 100%. In 3 tumor cell lines (Hela, A549 and U87), the pGL3-hTERT-Luc showed transcriptional activity equivalent to 13-21% of positive control activity, which was markedly higher than that of pGL3-basic plasmid (P<0.05). In contrast, there was no significant difference in transcriptional activity between the pGL3-hTERT-Luc and pGL3-basic plasmids in normal fibroblast cells (MRC5).

The article "Baculovirus Vector-Mediated Transfer of Sodium Iodide Symporter and Plasminogen Kringle 5 Genes for Tumor Radioiodide Therapy" was published in 2014. Journal: PLoS One.

**Figure 1:** Transcriptional activation induced by the hTERT promoter. The pGL3-hTERT-Luc, pGL3-Basic or pGL3-Control plasmids were co-transfected with pRL-SV40 plasmid into each cell line. The relative luciferase activity was determined. All data of firefly luciferase activity were corrected for renilla luciferase activity to account for variation in transfection efficiency and expressed as a percentage of results using the positive control. Each transfection was conducted in triplicate, and data represent the mean±sd.

### Expression of NIS gene in baculovirus-infected hela cells

The NIS gene in the baculovirus dual expression system was designed to be driven by the hTERT promoter for tumor-specific gene expression. As shown in Figure 2A, NIS mRNA expression levels were markedly increased in Hela cells but not in MRC5 cells after incubation with Bac-hTERT-NIS-Egr1-K5. By contrast, variably increased expression of NIS mRNA under control of the CMV promoter was observed in both cell lines. NIS protein expression was further confirmed by Western blotting analysis (Figure 2B). A band with a molecular mass of approximately 97 kDa recognized by the anti-NIS antibody was detected in lysates derived from Hela cells infected with Bac-hTERT-NIS-Egr1-K5 or Bac-CMV-NIS-Egr1-K5. In MRC-5 cells, the NIS protein band was only revealed after infection with Bac-CMV-NIS-Egr1-K5. These results indicated that tumor-specific expression of the NIS gene could be accomplished by hTERT promoter-based gene transfer.

**Figure 2:** Expression of NIS mRNA and protein in baculovirus-infected Hela cells. (A) Total RNA samples from baculovirus-infected Hela and MRC5 cells were extracted. NIS mRNA expression normalized to the GAPDH endogenous reference was detected by qRT-PCR. Results are expressed as means ± SD of three independent experiments. (B) Total cell lysates were prepared from Hela and MRC5 cells infected with recombinant baculovirus as described in Materials and Methods. NIS protein (∼97 kDa) expression was analyzed by Western blot, and GAPDH (∼36 kDa) was used as an internal control.

The article "Baculovirus Vector-Mediated Transfer of Sodium Iodide Symporter and Plasminogen Kringle 5 Genes for Tumor Radioiodide Therapy" was published in 2014. Journal: PLoS One.

### Expression of K5 gene in baculovirus-infected hela cells and HUVECs

The baculovirus dual expression system utilized another therapeutic gene, K5, under control of the Egr1 promoter to mediate radio-inducible K5 expression in proliferating endothelial cells. To identify the feasibility of radiosensitive Egr1 promoter and determine the optimal expression conditions, Hela cells were exposed to Na^131^I for different times or at different doses after incubation with Bac-hTERT-NIS-Egr1-K5. Western blotting of cell lysates using an anti-His-tag antibody showed a very weak expression of K5 protein (14 kDa) without irradiation and an elevated expression in a time-dependent manner with a peak level at 18 h after irradiation. Subsequently, dose-dependent K5 protein expression stimulated with Na^131^I for 18 h was identified. The K5 protein expression level was shown to be significantly elevated with irradiation (0∼20 MBq/mL) in infected Hela cells and highest at the dose of 5 MBq/mL (Figure 3A). However, the K5 protein expression began to decrease after irradiation for a longer time (30 h) or at a higher dose (20 MBq/mL). Thus, irradiation with Na^131^I at 5 MBq/mL for 18 h was determined to be the optimal dose for increasing expression of the K5 protein in the baculovirus-infected cells. These results were agreement with those of the qRT-PCR analysis (Figure 3B). Finally, the optimal condition of radio-inducible K5 expression was applied to HUVECs. Similarly, the K5 expression of baculovirus-infected HUVECs reached a peak at 18 h∼24 h after irradiation of 5 MBq/ml ^131^I (Figure 3C).

**Figure 3:** Expression of K5 mRNA and protein. (A) Time-dependent K5 protein (∼14 kDa) expression stimulated with 5 MBq/ml Na^131^I in Bac-hTERT-NIS-Egr1-K5-infected Hela cells was analyzed by Western blot. GAPDH was used as an internal control. Then Dose-dependent K5 protein expression stimulated with Na^131^I for 18 h in infected Hela cells was also extracted for Western blot analysis. (B) Total RNA samples from Hela cells were extracted after incubation with Bac-hTERT-NIS-Egr1-K5 and stimulation with or without 5 MBq/mL Na^131^I for 18 h. K5 mRNA expression normalized to the GAPDH endogenous reference was detected by qRT-PCR. Results are expressed as means ± SD of three independent experiments. *P<0.05. (C) Time-dependent K5 protein expression stimulated with 5 MBq/ml ^131^I in HUVECs infected with Bac-hTERT-NIS-Egr1-K5 was analyzed by Western blot. GAPDH was used as an internal control.

### Functional NIS activities in baculovirus-infected hela cells

The functional activity of the NIS protein was clearly shown by its cellular iodide uptake. As shown in Figure 4A, iodide uptake into Hela cells infected with Bac-hTERT-NIS-Egr1-K5 was rapid, reaching a maximum after approximately 30 min, followed by a decline. At 120 min after the addition of ^125^I, the uptake level was only 59.4% of peak activity. Hela cells infected with Bac-hTERT-NIS-Egr1-K5 showed up to a 5.6-fold increase in iodide accumulation, compared with that in cells co-incubated with perchlorate (P<0.05) after the incubation with ^125^I for 30 min (Figure 4B). No increase in iodide accumulation was observed in cells incubated with Bac-hTERT-0-Egr1-K5.

The article "Baculovirus Vector-Mediated Transfer of Sodium Iodide Symporter and Plasminogen Kringle 5 Genes for Tumor Radioiodide Therapy" was published in 2014. Journal: PLoS One.

**Figure 4:** In vitro iodide uptake in baculovirus-infected Hela cells. (A) Kinetics of ^125^I uptake. Bac-hTERT-NIS-Egr1-K5-infected Hela cells were incubated with Na^125^I at 37°C for 5∼120 min. Bac-hTERT-0-Egr1-K5 was used as a negative control. Results are expressed as means ± SD of three independent experiments. (B) Iodine perchlorate discharge test. Cells were incubated with ^131^I+30 μM sodium perchlorate or ^131^I alone. All experiments were performed in triplicate. (C) Cell survival rates after Na^131^I treatment. Baculovirus-infected Hela cells were incubated with Na^131^I at 5 MBq/mL for 18 h. Subsequently, cells were washed with bHBSS and incubated for 4 days. Cell survival was calculated as the percentage of absorbance relative to that in the blank group without ^131^I. Data are presented as means ± SD. *P<0.05.

Next, the in vitro therapeutic effect of radioiodine was estimated by determining the survival of cells in a cell proliferation assay using WST-8 dye. As shown in Figure 4C, the survival of Hela cells infected with Bac-hTERT-NIS-Egr1-K5 significantly decreased to 38.3%, when compared with those infected with Bac-hTERT-0-Egr1-K5 (76.0%) or non-infected cells (78.6%) (P<0.05). These observations suggested that tumor cells could be effectively and specifically killed by NIS-mediated uptake of^ 131^I.

### Apoptotic effect of ^131^I-stimulated K5 in baculovirus-infected HUVECs

We next investigated the therapeutic efficacy of the ^131^I-stimulated apoptotic effect of K5 in HUVECs. In HUVECs infected with Bac-hTERT-NIS-Egr1-K5, the percentage of early apoptotic cells markedly increased to 30.8% compared with those infected with Bac-hTERT-NIS-Egr1-0 (11.2%) and non-infected cells (10.9%) (Figure. 5). These results demonstrated that ^131^I could induce the K5-based apoptotic effect in HUVECs.

**Figure 5:** Early apoptotic effects of ^131^I-induced K5 in HUVECs. Baculovirus-infected HUVEC cells were incubated with Na^131^I at 5 MBq/mL for 18 h, followed by analysis using the Annexin V-FITC Apoptosis Detection Kit. Percentages of early apoptotic cells are expressed as means ± SD.*P<0.05.

The article "Baculovirus Vector-Mediated Transfer of Sodium Iodide Symporter and Plasminogen Kringle 5 Genes for Tumor Radioiodide Therapy" was published in 2014. Journal: PLoS One.

### ^131^I imaging of tumor xenografts and quantification

To noninvasively monitor the successful transfer of therapeutic genes into tumors, NIS gene-based ^131^I imaging was perfomed by SPECT. When the diameter of Hela tumor xenografts reached up to 5-8 mm, whole-body scintigraphic imaging was performed on the mice by SPECT after injection of ^131^I at 7.4 MBq via the tail vein. In contrast to negative control tumors, which showed negligible uptake of ^131^I, tumors infected with Bac-hTERT-NIS-Egr1-K5 showed significant uptake, indicating functional NIS expression (Figure 6A). Physiologic uptake was also observed in the stomach where NIS is normally expressed and in the bladder as the path of ^131^I excretion. Regions of interest were drawn on the images of the tumors, and ^131^I activity in those tumors was quantified at various time points (Figure 6B). The accumulation of ^131^I in tumors reached a maximum level at 0.5 h, followed by a rapid decline (half-life, 3.2 h). By 16 h, the accumulation had decreased to 1.76%ID/g, similar to the negative control.

**Figure 6:** In vivo tumor scintigraphic imaging and changes in tumor volume. (A) Mice were subcutaneously transplanted with Hela cells in the right axilla (A3). SPECT images at 0.5 h post-injection with Na^131^I showed that the tumor was clearly visualized in the baculovirus-infected group (A2) but not in the PBS group (A1). (B) ^131^I accumulation in tumors over time. Regions of interest in the tumor were quantified and expressed as means ± SD. (C) Changes in tumor volumes after ^131^I treatment. Twenty-four hours after intratumoral injection with recombinant baculovirus or PBS, the mice were further injected with 37 MBq of Na^131^I via the tail vein. Data are presented as means ± SD. *P<0.05.

### Inhibitory effect of ^131^I on baculovirus-infected tumor growth in vivo

Athymic nude mice-bearing Hela tumors were randomly divided into three treatment groups and injected with Bac-hTERT-NIS-Egr1-0+^131^I, Bac-hTERT-0-Egr1-K5+^131^I or Bac-hTERT-NIS-Egr1-K5+^131^I (Figure 6C). Two groups of mice treated with PBS alone or PBS+^131^I served as control groups. Prior to therapy, no significant difference was found in the tumor volume among the five groups. All tumor volumes in the five groups increased gradually during follow-up. Fifteen days after 37 MBq ^131^I treatment, Bac-hTERT-NIS-Egr1-K5-infected tumors showed a significant growth retardation compared to control groups or the other two treated groups (P<0.05). Unfortunately, treatment with Bac-hTERT-0-Egr1-K5+^131^I or Bac-hTERT-NIS-Egr1-0+^131^I showed no significant effect on tumor growth compared to the control groups. These results demonstrated that the combination of radioiodide and antiangiogenesis therapy could enhance the anti-tumor effects in vivo.

The article "Baculovirus Vector-Mediated Transfer of Sodium Iodide Symporter and Plasminogen Kringle 5 Genes for Tumor Radioiodide Therapy" was published in 2014. Journal: PLoS One.

### Immunohistological analysis of tumors

To further confirm the effect of ^131^I-stimulated K5 on tumor neovascularization, we performed histological analysis on the dissected tumors (Figure 7). CD31 staining was carried out by quantitatively analyzing the MVD in tumors. CD31-immunostained microvessels were found to be markedly decreased in the Bac-hTERT-NIS-Egr1-K5+^131^I group compared to the control groups (P<0.05). Treatment with Bac-hTERT-0-Egr1-K5+^131^I also reduced the number of tumor microvessels compared to the control groups (P<0.05). Therefore, these results indicated that ^131^I-induced K5 therapy was effective against Hela xenografts in the mouse model.

**Figure 7:** Immunohistochemical staining of CD31 and MVD determination. (A) Immunohistochemical staining with anti-CD31 antibody. The arrow indicates a representative microvessel within the tumor (magnification, 400×). (B) MVD was determined by identifying the three most intense areas of neovascularization of each sample and counting at low power (magnification, 100×). Average vessel counts of the three selected fields were recorded.*P<0.05.

## Discussion

Angiogenesis has been demonstrated to be important for the growth and survival of tumor cells, suggesting that both tumor cells and their supporting endothelial cells should be considered for targeted cell killing when designing cancer treatments [20]. NIS has been widely investigated as a potential therapeutic gene for cancer. Transfer of the NIS gene into a variety of tumors, including cervical cancer [21], breast cancer [22] and prostate carcinoma [23], has shown the capacity to confer radioiodide uptake. Although intracellular iodine is rapidly released, resulting in limited retention time of the radioiodide within cells, NIS-based radioiodide therapy has demonstrated therapeutic efficacy in vitro and in partial tumor xenograft studies. The NIS gene is also well known for its advantages as a reporter gene. In the present study, ^131^I SPECT revealed a clear image of recombinant baculovirus-infected tumors in vivo, and the uptake of ^131^I in tumors could be quantified. These results suggest that the NIS gene would be a useful tool to allow noninvasive monitoring of vector-mediated gene expression in vivo.

Specificity is an important concept for cancer gene therapy. A specific promoter can restrict expression of the NIS gene only in target cells and reduce unnecessary radioiodide uptake in normal tissues. Several groups have demonstrated good responses to NIS-based radioiodide therapy in various tumors using tissue-specific promoters, including those for prostate-specific antigen [24], carcinoembryonic antigen [25] and calcitonin [26]. However, the hTERT promoter would be useful for gene therapy for a wide range of cancers. In our study, a much higher transcriptional activity of the hTERT promoter was demonstrated in tumor cells than that in normal cells. Previous studies showed that targeted expression of a therapeutic transgene such as NIS and caspase-8 can be achieved under control of the hTERT promoter [6], [27]. However, specific promoters often exhibit lower activity levels than those of non-specific ones such as the CMV promoter. We found that the expression of NIS under the hTERT promoter was similar to that from the CMV promoter. The iodide uptake assay also demonstrated that a robust and functional NIS activity could be mediated by the hTERT promoter. Thus, the hTERT promoter may provide not only specificity but also a relatively strong transcriptional activity for targeted gene expression.

The article "Baculovirus Vector-Mediated Transfer of Sodium Iodide Symporter and Plasminogen Kringle 5 Genes for Tumor Radioiodide Therapy" was published in 2014. Journal: PLoS One.

K5 as an antiangiogenic agent exerts its effect on endothelial cells by inducing cell cycle arrest. In preclinical and clinical trials, however, investigations of antiangiogenic agents have indicated that tumor cures are limited when these agents are used as the sole method of treatment [28]. Further preclinical studies suggest that the combination of radiotherapy and angiogenic blockade enhances the therapeutic success of ionizing radiation by targeting both tumor cells and tumor vessels [7], [29]. Thus, the antiangiogenic therapy combined with radionuclide therapy was anticipated as a potential method for enhancing the antitumor effect. In the present study, Bac-hTERT-NIS-Egr1-K5 showed a significant ^131^I-induced killing effect in tumor cells and an apoptotic effect in endothelial cells in vitro. And the efficacy of the therapeutic strategy was further validated in vivo.

To ensure the spatial and temporal synchronism of ^131^I radiation in tumor cells and K5-induced apoptosis in endothelial cells, the radiation-inducible Egr1 promoter was inserted in our recombinant baculovirus dual expression vector. We found that ^131^I could activate the Egr1-mediated K5 expression in a dose and time-dependent manner in vitro. Thus, radioiodine could serve as a switch to simultaneously activate the two therapeutic pathways from this vector system. The potential advantage of radiation-inducible genetic constructs has been demonstrated in the so-called “genetic radiotherapy” strategy. A preclinical study has shown that tumors infected with a replication-defective adenovirus carrying the TNF-α gene under control of the Egr1 promoter could respond to radiotherapy with local production of TNF-α and substantial increases in anti-tumor activity, without toxicities encountered when this cytokine was administrated systemically [29]. However, radiotherapy is often unsuitable for the treatment of multiple metastatic lesions. The use of radioisotopes that accumulate in tumors offers an advantage for selective induction of exogenous genes.

The article "Baculovirus Vector-Mediated Transfer of Sodium Iodide Symporter and Plasminogen Kringle 5 Genes for Tumor Radioiodide Therapy" was published in 2014. Journal: PLoS One.

Utilizing radioiodine and antiangiogenic therapy together may be a useful strategy for cancer therapy, but the mechanism underlying the effects of this combination is presently unclear. Oxygen is known to be a potent radiosensitizer and, through interaction with the radicals formed by radiation, is essential for the induction of radiation-induced DNA damage. Abnormalities in the tumor neovasculature often induce increased interstitial pressure (IP) and further reduce perfusion and oxygenation of tumor cells, leading to radiation resistance. Antiangiogenic therapy may temporarily “normalize” the existing tumor vasculature [30] by lowering the IP and improving perfusion and oxygenation, thus increasing sensitivity of tumor cells to ionizing radiation.

However, it should be noted that although there was a statistically significant difference in tumor volume, Bac-hTERT-NIS-Egr1-K5-treated tumors grew exponentially. The lack of sustained growth arrest may be due to the relatively low infection efficiency of the baculovirus. As an insect virus in nature, baculovirus does not replicate inside the transduced cells, and its DNA degrades in the cells over time. Therefore, its infectivity for mammalian cells is relatively weak and the duration of expression of virus production is short. In our study, the amount of baculovirus was likely to be not enough in a single injection for supporting a sustained gene expression. So multiple virus injections with a repeated administration of^ 131^I may overcome this problem. In addition, previous studies have indicated that baculovirus-mediated transgene expression could be elevated by the supplementation of histone deacetylase (HDAC) inhibitors [31] or by modifying the envelope protein of baculovirus such as vesicular stomatitis virus G (VSVG) protein [32].

Although further applications of baculovirus have been hampered by a number of bottlenecks, including fragile nature of virus and serum complement inactivation in vivo, baculovirus is still a promising gene delivery vector due to its advantages such as low toxicity, huge cloning capacity and production convenience.

## Conclusion

We have developed a baculovirus dual expression vector which contains the NIS gene under the control of a tumor-specific promoter, hTERT, and the K5 gene driven by a radiation-inducible promoter, Egr1. Its therapeutic effects were validated in vitro on cervical cancer cells and endothelial cells. In vivo, ^131^I SPECT imaging revealed a clear image of the tumor xenografts, and therapeutic experiments with ^131^I in baculovirus-infected tumors further confirmed the potential of this new strategy of NIS-mediated gene therapy accompanied by K5-based antiangiogenic therapy.
